# Automated COVID-19 Classification Using Heap-Based Optimization with the Deep Transfer Learning Model

This article has been retracted.

**DOI:** 10.1155/2022/7508836

**Published:** 2022-08-22

**Authors:** Bahjat Fakieh, Mahmoud Ragab

**Affiliations:** ^1^Information Systems Department, Faculty of Computing and Information Technology, King Abdulaziz University, Jeddah 21589, Saudi Arabia; ^2^Information Technology Department, Faculty of Computing and Information Technology, King Abdulaziz University, Jeddah 21589, Saudi Arabia; ^3^Department of Mathematics, Faculty of Science, Al-Azhar University, Naser City 11884, Cairo, Egypt; ^4^Centre for Artificial Intelligence in Precision Medicines, King Abdulaziz University, Jeddah 21589, Saudi Arabia

## Abstract

The outbreak of the COVID-19 pandemic necessitates prompt identification of affected persons to restrict the spread of the COVID-19 epidemic. Radiological imaging such as computed tomography (CT) and chest X-rays (CXR) is considered an effective way to diagnose COVID-19. However, it needs an expert's knowledge and consumes more time. At the same time, artificial intelligence (AI) and medical images are discovered to be helpful in effectively assessing and providing treatment for COVID-19 infected patients. In particular, deep learning (DL) models act as a vital part of a high-performance classification model for COVID-19 recognition on CXR images. This study develops a heap-based optimization with the deep transfer learning model for detection and classification (HBODTL-DC) of COVID-19. The proposed HBODTL-DC system majorly focuses on the identification of COVID-19 on CXR images. To do so, the presented HBODTL-DC model initially exploits the Gabor filtering (GF) technique to enhance the image quality. In addition, the HBO algorithm with a neural architecture search network (NasNet) large model is employed for the extraction of feature vectors. Finally, Elman Neural Network (ENN) model gets the feature vectors as input and categorizes the CXR images into distinct classes. The experimental validation of the HBODTL-DC model takes place on the benchmark CXR image dataset from the Kaggle repository, and the outcomes are checked in numerous dimensions. The experimental outcomes stated the supremacy of the HBODTL-DC model over recent approaches with a maximum accuracy of 0.9992.

## 1. Introduction

COVID-19 is a renowned communicable disease caused by severe acute respiratory syndrome coronavirus 2 (SARS-CoV-2) that is regarded as a coronavirus strain. Given the hike in new COVID-19 cases and the reopening of everyday routines throughout the universe, the demand for curtailing the epidemic is highly highlighted. Artificial intelligence (AI) and medical images were noted to be very helpful for speedy valuation to render medication for COVID-19 victims [2]. Thus, the placement and model of AI apparatus for image categorization of COVID-19 in a shorter span with confined data is an emergency requirement for combating the present epidemic. Radiotherapists have currently discovered deep learning (DL) advanced in AI that could identify tuberculosis in chest X-rays (CXR), help detect lung aberrations relevant to COVID-19, and aid doctors in determining the dosage of medication for high-risk coronavirus infected victims [3]. The medical imaging task was verified by others which acted as a vital resource of information to permit the speedy prognosis of COVID-19, and the joining of chest imaging and AI might be helpful in describing the complexities of COVID-19.

Since AI could find paradigms in CXR which are usually not identified by radiotherapists [4], there are several studies stated in literature regarding the latest advancements in DL techniques by employing convolutional neural networks (CNNs) for distinguishing COVID-19 and non-COVID-19 with the help of public databases of CXR (relevant studies were provided in the following segment) [5]. CNN is one of the more familiar methodologies in AI in the present era. CNN has been successfully used in in medical image analysis such as ultrasonography, MRI, CT scans, and X-ray. CNN is more successful in speech recognition, natural language processing (NLP), audio recognition, and computer vision. Additionally, a neural network (NN) is a sequence of methods which identifies relations in datasets via a process which is more identical to human brain function [6]. This method is highly efficient for image processing and pattern recognition. It gets images as input and constructs a design which operates on the images to derive the features from those images and identify a paradigm. CNN recognizes the resemblances of new inputs as exactly as possible by utilizing the pattern. This system became famous due to its simpler form and decreased training variables, low complexity, and adaptability of the network system [7].

COVID-19 recognition with the help of CNN is a well-accomplished research method once it turns out to be a global pandemic. We have discovered marvelous CNN-related research studies with the use of CT scan images along with X-ray images to notice and categorize COVID-19 [8]. However, such CNN approaches have produced splendid resultants; it is not considered an alternate to definite testing approaches so far. These systems seem to be useful in accordance with definite testing methodologies, but then there exists a large chamber for research and enhancement before commercial usage [9]. A great number of data scientists and researchers are putting their efforts into creating more precise and dependable deep learning-related identification methods for recognizing COVID-19. The author's main focus is on DL methods to indicate features from CT and X-ray images of coronavirus-infected patients [10].

This study develops a Heap-based Optimization with Deep Transfer Learning model for detection and classification (HBODTL-DC) of COVID-19. The proposed HBODTL-DC model uses the Gabor filtering (GF) method to improve the image quality. Besides, the HBO algorithm with a neural architecture search network (NasNet) large model is utilized as a feature extractor. At last, Elman Neural Network (ENN) technique receives the feature vectors as input and categorizes the CXR images into distinct classes. The experimental validation of the HBODTL-DC model takes place on benchmark CXR image datasets, and the outcomes are inspected under numerous dimensions.

## 2. Related Works

This section performs a brief evaluation of recently developed COVID-19 recognition models. In [11], DL-based techniques such as deep feature extracting, fine tuning of pre-trained CNN, and endwise trained of the established CNN method are utilized for classifying COVID-19 and normal (healthy) chest X-ray images. In order to perform deep feature extraction, pre-trained deep CNN (DCNN) techniques (VGG16, ResNet18, ResNet50, VGG19, and ResNet101) are utilized. In order to classify deep features, the SVM classification was utilized with several kernel functions such as Gaussian, linear, quadratic, and cubic. In [12], a detailed estimation of eight pre-trained techniques is projected. The testing, training, and validating of these techniques are executed on chest X-ray (CXR) images going to five various classes, comprising an entire 760 images. In the fine-tune techniques, pre-trained from the ImageNet dataset are computationally effectual and accurate.

Khan et al. [13] present CoroNet, a DCNN technique, for automatically identifying COVID-19 infection in the chest X-ray image. The presented technique was dependent upon Xception structure and pre-trained on the ImageNet dataset and trained endwise on a dataset organized by gathering COVID-19 and other chest pneumonia X-ray images in 2 distinct publicly accessible databases. Basu et al. [14] examine a novel model named “domain extension transfer learning” (DETL). Used DETL, with pre-trained DCNN, on a compared huge chest X-ray dataset, is tuned to classify amongst 4 classes using COVID-19: normal, pneumonia, and other disease. A 5-fold cross-validation was executed to estimate the possibility of utilizing CXR for analyzing COVID-19. Ahsan et al. [15] presented a machine vision technique for detecting COVID-19 in the chest X-ray image. The feature extraction by CNN and histogram-oriented gradient (HOG) in X-ray images is merged for developing the classifier method with training by CNN (VGGNet). The modified anisotropic diffusion filtering (MADF) approach is utilized for optimum edge preservation and to decrease noise in the images. The watershed segmentation technique has been utilized for marking the important fracture area from the input X-ray images.

Sakib et al. [16] presented a possible and effectual DL-related chest radiograph classification (DL-CRC) structure for distinguishing the COVID-19 case having higher accuracy in any other abnormal (for instance, pneumonia) and regular cases. In [17], the authors established an Auxiliary Classifier Generative Adversarial Network (ACGAN) for generating CXRs. All the generated X-rays point to two classes of COVID-19: positive or normal.

## 3. The Proposed Model

In this study, a new HBODTL-DC technique was enhanced for the identification of COVID-19 on CXR images. The presented HBODTL-DC model incorporates GF preprocessing, NASNetLarge feature extraction, HBO-related hyperparameter optimization, and ENN-related classification. The design of the HBO algorithm supports ineffectual choice of hyperparameters related to the NASNetLarge model, which in turn considerably improves the classifier results.  Figure 1 depicts the block diagram of the HBODTL-DC approach.

### 3.1. GF-Based Preprocessing

The GF model is beneficial to enhancing the image as a result of its ability to select direction and tune to a particular frequency. It is chosen over other filters due to the fact that it is highly flexible in the definition of the function shape. We adapted the 2D-GF for the contrast enhancement of retinal images in the frequency domain [18]. A continuous WT,  *T*_*ψ*_(*b*,  *θ*,  *a*), can be defined by the scalar product of the image *I* with the transformed wavelet *ψ*_*b*,*θ*,*a*_ as

(1) $$\begin{array}{c} T_{\psi }\left(b,\theta ,\;a\right)=C_{\psi }^{-1/2}\langle \psi_{b,\theta ,a}|I\rangle ,\\ =C_{\psi }^{-1/2}a^{-1}\int \psi^{*}\left(a^{-1}r_{-\theta }\left(x-b\right)\right)I\left(x\right){\text{d}}^{2}x. \end{array}$$

Let *ψ* be the analyzing wavelet, *ψ*^*∗*^ denote the complex conjugate of *ψ*, and *C*_*ψ*_ indicate the normalized constant. The parameters , *θ*  and  *b* represent the dilation scale, rotation angle, and displacement vector, correspondingly. *r*_*θ*_ indicates the rotation operator act on *x* = (*x*, *y*), that is determined by

(2) $$\begin{array}{c} r_{\theta }\left(x\right)=\left(x\;\cos\;\theta -y\;\sin\;\theta ,\;x\;\sin\;\theta +y\;\cos\;\theta \right),\;0\leq \theta \leq 2\pi . \end{array}$$

The 2D-GF is designated by the analyzing wavelet:

(3) $$\begin{array}{c} \psi \left(x\right)=\exp\left(jkx\right)\exp\;\left(-\frac{1}{2}{\left|Ax\right|}^{2}\right). \end{array}$$

The *η* parameter is crucial because small values have lesser effects on the vessel enhancement, and large values generate a longer width of the retinal vessel. Consequently, we fixed *η* as a 4. Examine the maximum contrast between background and vessels, the magnification level of retinal image transformation, along with constraining the intensity amplification of nonvessel pixels. For all the pixels, we extracted the maximal response over each potential orientation with preferred scale values. The outcome of GF is represented as follows:

(4) $$\begin{array}{c} M_{\psi }\left(b,\;a\right)=\;\underset{\theta }{\max}\left|T_{\psi }\left(b,\;\theta ,\;a\right)\right|, \end{array}$$

where *θ* indicates the angle ranges from 0° to 170°, with a step of 10°.

### 3.2. Feature Extraction

Once the input CXR images are preprocessed, the next phase is to produce feature vectors via the NASNetLarge model. CNN is a type of FFNN model that has better outcomes in natural language processing (NLP) and image processing. It is efficiently employed in the calculation of sequential time. The weight sharing and local perception of CNN might considerably decrease the parameter number, therefore enhancing the efficacy of the learning model. CNN is primarily comprised of full connection, convolution, and pooling layers. All the convolutional layers comprise a variety of convolutional kernels, and their computation can be demonstrated by the following expression. Afterward, from the convolutional process of the convolutional layer, the feature of the information is extracted. However, the extracted feature dimension is higher. Hence, to resolve the challenge and decrease the cost of network training, a pooling layer is included after the convolutional layer for decreasing the feature dimension:

(5) $$\begin{array}{c} l_{t}=\tanh\left(x_{t}*k_{t}+b_{t}\right), \end{array}$$

where *l*_*t*_ indicates the output afterward convolutional layer, tanh indicates the activation function, *x*_*t*_ denotes the input vector, *k*_*t*_ represents the weight of the convolutional kernel, and *b*_*t*_ denotes the bias of the convolutional kernel. TL is a DL method that employs a pre-trained model on larger datasets for initializing a trained model on dissimilar datasets. CNN tends to perform well with large datasets when compared to small ones. TL is effective in CNN applications in which the datasets are smaller. In recent times, TL has been utilized for detecting objects, image classification, and medical imaging. A model trained on larger datasets such as ImageNet is utilized as a feature extractor for applications with small datasets such as the brain MRI dataset. The advantages of TL are the fast training process, prevention of overfitting, training with less information, and better efficiency. The pre-trained CNN method utilized is the NASNetLarge method.

NASNet is a model constructed by a neural structure searching algorithm [19]. This concept is realized using the NAS concept proposed by the Google ML team. The technique depends on reinforcement learning. Here, the efficacy of the child block is checked by the parental block, and the structure of the neural network is tuned. Some variations have been taken place according to optimizer function, weight, regularization method, and so on, for improving network's efficiency. The system component includes a CNN block and a recurrent controller neural network (CRNN). A block is the small element of the NASNet structure, and a cell is an integration of blocks. The network searching space can be constructed by separating the networks into cells and additionally dividing them into blocks. Probable operations for blocks involve identity mapping, separable convolution, regular, and pooling convolutions. At present, the NasNet method is designated for identifying COVID-19 and non-COVID-19 patients since the system has an accessible structure for classifying images and is comprised of reduced and normal cells.

### 3.3. Hyperparameter Optimization

In order to effectually modify the hyperparameters related to the NASNetLarge method, the HBO algorithm is exploited. Qamar et al. [20] suggested a latest MH named HBO, viz., motivated by the employee's responsibilities and job description titles. The corporate rank hierarchy (CRH) is regarded as the general framework applied mostly in corporations. HBO is determined by four major stages: (1) interaction with the immediate boss, (2) CRH, (3) employee self-contribution, and (4) interaction among colleagues.In the following, the HBO stages are mathematically modeled.

CRH: it is modeled by the heap data structure. In the heap, the searching agent fitness can be determined by the index of the searching agent, and the key node in the population is determined as the value of the node in the heap.

Interaction with immediate boss: in general, the upper levels of the central organizing framework are accountable to impose restriction and policies; thus, the subordinate (children) follows the immediate boss (parental node). For modeling those behaviors, the location of every searching agent ${\overset{⟶}{x}}_{i}$ would be upgraded based on the parental node B in the following:

(6) $$\begin{array}{c} X_{i}^{k}\left(t+1\right)=B^{k}+\gamma \lambda^{k}\left|B^{k}-X_{i}^{k}\left(t\right)\right|. \end{array}$$

From the expression, the present iteration is represented as *r*, the *k*, th components of a vector are characterized as follows [21], And the variable *λ*^*k*^ indicates the component of vector. $\overset{⟶}{\lambda }$ is evaluated according to the arbitrary value within (*r* *in* [0,1]) as

(7) $$\begin{array}{c} \overset{⟶}{\lambda }=2r-1. \end{array}$$

In (7), the variable *γ* is determined in (6) and is evaluated by

(8) $$\begin{array}{c} \gamma =\left|2-\frac{\left(t\mathrm{mod}\;T/c\right)}{T/4c}\right|, \end{array}$$

where *C* and *T* symbolize designed variable and the max amount of iterations, correspondingly. In general, *γ* linearly decreases from 2 to 0.

Interaction between colleagues: in HBO, the colleagues are agents, and the location of every agent $\overset{⟶}{x}$ can be upgraded by their random colleague ${\overset{⟶}{S}}_{r}$ as follows:

(9) $$\begin{array}{c} \chi_{i}^{k}\left(t+1\right)=\left\{\begin{array}{cc} S_{r}^{k}+\gamma^{\lambda^{k}}\left|S_{r}^{k}-X_{i}^{k}\left(t\right)\right|, & f\left({\overset{⟶}{s}}_{r}\right)<f\left({\overset{⟶}{x}}_{i}\left(t\right)\right),\\ x_{i}^{k}+\gamma^{\lambda^{k}}\left|S_{r}^{k}-x_{i}^{k}\left(t\right)\right|, & f\left({\overset{⟶}{S}}_{r}\right)\geq f\left({\overset{⟶}{x}}_{i}\left(t\right)\right), \end{array}\right) \end{array}$$

where the aim of the objective function(*f*) is to evaluate fitness of the searching agent. When $\left({\overset{⟶}{S}}_{r}\right)<f\left({\overset{⟶}{x}}_{i}\left(t\right)\right)$, (9) aims at allowing the searching agents to search the region around (*S*_*r*_^′〈^) or else, around *x*_*i*_.

Employee's self-contribution: here, the self-contribution can be implemented by storing the preceding employee's location as

(10) $$\begin{array}{c} x_{i}^{k}\left(t+1\right)=x_{i}^{k}\left(t\right). \end{array}$$

A roulette wheel is employed to separate the population into *p*_1_, *p*_2_, and *p*_3_ proportions for maintaining the balance between exploitation and exploration, *p*_1_ permits a searching agent to upgrade the location. Furthermore, *p*_1_, *p*_2_, and *p*_3_ proportions are evaluated as follows, where *t* describes the existing iteration and *T* indicates the maximal amount of iterations:

(11) $$\begin{array}{c} p_{1}=1-\frac{t}{T},\\ p_{2}=p_{1}+\frac{1-p_{1}}{2},\\ p_{3}=p_{2}+\frac{1-p_{1}}{2}=1. \end{array}$$

To summarize, a common method for upgrading the searching agent position is given by

(12) $$\begin{array}{c} X_{i}^{k}\left(t+1\right)=\left\{\begin{array}{c} X_{i}^{k}\left(t\right),\;p\leq p_{1}\\ B^{k}+\gamma \lambda^{k}\left|B^{k}-x_{i}^{k}\left(t\right)\right|,\;p>p_{1}\;,\;p\leq p_{2}\\ S_{r}^{k}+\gamma \lambda^{k}\left|S_{r}^{k}-x_{i}^{k}\left(t\right)\right|,\\ p>p_{2}\;,\;p\leq p_{3},\;f\;\left({\overset{⟶}{S}}_{r}\right)<f\left({\overset{⟶}{x}}_{i}\left(t\right)\right)\\ X_{i}^{k}+\gamma \lambda^{k}\left|S_{r}^{k}-X_{i}^{k}\left(t\right)\right|,\\ p>p_{2},\;p\leq p_{3}\;,\;f\;\left(\overset{⟶}{S}\right)\geq f\left({\overset{⟶}{x}}_{i}\left(t\right)\right) \end{array}\right), \end{array}$$

where *p* in [0,1] indicates an arbitrary number. It is worth mentioning here that (6) boosts convergence and exploitation, (10) increases exploration, and (9) endorses exploration and exploitation.

The HBO system advances a fitness function (FF) for obtaining higher classifier performances. It describes a positive integer to signify the best performances of candidate solutions. Throughout this case, the minimized classifier error rate has been regarded as FF as presented in

(13) $$\begin{array}{c} \text{fitness}\left(x_{i}\right)=\text{Classifier Error Rate}\left(x_{i}\right)\\ =\frac{\text{number of misclassified samples}}{\text{Total number of samples}}*100. \end{array}$$

### 3.4. Image Classification

In the final stage, the ENN model is applied to categorize the CXR images into distinct classes. The ENN method encompasses input, context, output, and hidden layers. The main configuration of the ENN mechanism is comparable to the FFNN in that the connections excepting context layers are similar to MLP [22]. The context layer gets the input from the output of the hidden state for storing the early value of the hidden state. The output weight, external input, and context weight matrixes are characterized by *W*_*h*_^*i*^, *W*_*h*_^*c*^, and *W*_*h*_^0^, respectively. The dimension of the output and input layers are represented as *n*, viz., the dimension of the context layer is *m*  and *x*^1^(*t*)=[*x*_1_^1^(*t*), *x*_2_^1^(*t*),…,*x*_*n*_^1^(*t*)]^*T*^ and *y*(*t*)=[*y*_1_(*t*),  *y*_2_(*t*),  …,  *y*_*n*_(*t*)]^*T*^.

The input unit of ENN mechanism is determined by the following equation:

(14) $$\begin{array}{c} u_{i}\left(l\right)=e_{i}\left(l\right),\;\;i=1,2,\;\ldots ,\;n, \end{array}$$

where *l* determines the input and output units at *l* round. Then, the *k*, th hidden state in the network is characterized as follows:

(15) $$\begin{array}{c} v_{k}\left(l\right)=\sum_{j=1}^{N}\omega_{kj}^{1}\left(l\right)x_{j}^{c}\left(l\right)+\sum_{i=1}^{n}\omega_{ki}^{2}\left(l\right)u_{i}\left(l\right),\\ k=1,2,\;\ldots ,\;N, \end{array}$$

where *x*_*j*_^*c*^(*l*) describes the signal that is distributed from the *k*, th context nodes and *ω*_*kj*_^1^(*l*) defines *i*, th and *j*, th weights of the hidden states directed from *o*, th  nodes. Finally, the outcomes of the hidden state are fed into the context layers as shown in the following:

(16) $$\begin{array}{c} W_{k}\left(l\right)=f_{0}\left({\bar{v}}_{k}\left(l\right)\right). \end{array}$$

Here,

(17) $$\begin{array}{c} {\bar{v}}_{k}\left(l\right)=\frac{v_{k}\left(l\right)}{\max\left\{v_{k}\left(l\right)\right\}}. \end{array}$$

The above equation signifies the normalized values of the hidden state. The subsequent layers represent the context layer that is determined:

(18) $$\begin{array}{c} C_{k}\left(l\right)=\beta C,\left(l-1\right)+W_{k}\left(l-1\right),\;\;k=1,2,\;\ldots ,\;N, \end{array}$$

where *W*_*k*_ indicated the gain of self-connected feedback amongst [0, 1]. Finally, the output unit at the network is characterized as

(19) $$\begin{array}{c} y_{0}\left(l\right)=\sum_{k=1}^{N}\omega_{ok}^{3}\left(l\right)W_{k},\left(l\right),\;\;0=1,2,\text{ …},\;n, \end{array}$$

where *ω*_*ok*_^3^ determines the weight of the connection from *k*, th layers into the *o*, th layers.  Figure 2 illustrates the framework of the ENN.

## 4. Results and Discussion

This section assesses the COVID-19 classification results of the HBODTL-DC model on the benchmark dataset from the Kaggle repository [23]. The dataset holds images under four classes, namely, COVID-3616, Lung_Opacity-6012, Normal-10192, and Viral Pneumonia-1345. In this study, we have taken a set of 3224, 3224, and 1345 samples under COVID-19, normal, and pneumonia classes, respectively. A few sample images are depicted in Figure 3. The parameter settings are given as follows: learning rate, 0.01, dropout, 0.5, batch size, 5, epoch count, 50, and activation, ReLU.

Figure 4 exhibits a brief set of confusion matrices offered by the HBODTL-DC model on test data. With run-1, the HBODTL-DC model has recognized 3204, 3180, and 1336 images into COVID-19, healthy, and viral pneumonia classes, respectively. Along with that, with run-2, the HBODTL-DC methodology has recognized 3208, 3192, and 1336 images into COVID-19, healthy, and viral neumonia classes, correspondingly. Afterward, with run-4, the HBODTL-DC approach has recognized 3223, 3221, and 1340 images into COVID-19, healthy, and viral pneumonia classes, correspondingly. At last, with run-5, the HBODTL-DC algorithm has recognized 3220, 3218, and 1338 images into COVID-19, healthy, and viral pneumonia classes, correspondingly.

Table 1 and Figure 5 display the overall classifier outcomes of the HBODTL-DC model on the test data under five distinct runs. The obtained results implied that the HBODTL-DC model has demonstrated improved results under every run. For instance, on run-1, the HBODTL-DC model has provided an average accu_*y*_, prec_*n*_, sens_*y*_, spec_*y*_, and *F*_score_ of 99.38%, 98.80%, 99.12%, 99.54%, and 98.95%, respectively. Meanwhile, on run-3, the HBODTL-DC system has offered an average accu_*y*_, prec_*n*_, sens_*y*_, spec_*y*_, and *F*_score_ of 99.72%, 99.34%, 99.66%, 99.81%, and 99.49%, correspondingly. Eventually, on run-4, the HBODTL-DC approach has provided an average accu_*y*_, prec_*n*_, sens_*y*_, spec_*y*_, and *F*_score_ of 99.92%, 99.91%, 99.83%, 99.93%, and 99.87%, correspondingly. Concurrently, on run-1, the HBODTL-DC algorithm has obtained an average accu_*y*_, prec_*n*_, sens_*y*_, spec_*y*_, and *F*_score_ of 99.85%, 99.80%, 99.72%, 99.88%, and 99.76%, correspondingly.

A brief precision-recall examination of the HBODTL-DC model on test dataset is represented in Figure 6. By observing the figure, it is noticed that the HBODTL-DC model has accomplished maximum precision-recall performance under all classes.

A detailed ROC investigation of the HBODTL-DC model on test dataset is exhibited in Figure 7. The results indicated that the HBODTL-DC approach has exhibited its ability in categorizing three different classes such as COVID, healthy, and viral pneumonia on the test dataset.

The training accuracy (TA) and validation accuracy (VA) attained by the HBODTL-DC methodology on test dataset is demonstrated in Figure 8. The experimental outcome represents that the HBODTL-DC algorithm has gained maximum values of TA and VA. In specific, the VA seemed to be higher than TA.

The training loss (TL) and validation loss (VL) achieved by the HBODTL-DC system on test dataset are established in Figure 9. The experimental outcome inferred that the HBODTL-DC approach has accomplished least values of TL and VL. In specific, the VL seemed to be lower than TL.

Table 2 and Figure 10 report a detailed comparative examination of the HBODTL-DC model with recent models on CXR images [24–26]. The results indicated that the HBODTL-DC model has gained maximum performance over other models. With respect to sens_*y*_, the HBODTL-DC model has offered improved sens_*y*_ of 0.9983, whereas the DBHL, DHL-2, DHL-1, ResNet-2, TL-ResNet-2, ResNet-1, TL-RENet-1, and QSGOA-DL models have obtained reduced sens_*y*_ values of 0.9900, 0.9900, 0.9800, 0.9700, 0.9800, 0.9700, 0.9700, and 0.9972, respectively. In addition, in terms of spec_*y*_, the HBODTL-DC technique has presented higher spec_*y*_ of 0.9993, whereas the DBHL, DHL-2, DHL-1, ResNet-2, TL-ResNet-2, ResNet-1, TL-RENet-1, and QSGOA-DL approaches have gained decreased spec_*y*_ values of 0.9800, 0.9700, 0.9800, 0.9700, 0.9800, 0.9700, 0.9900, and 0.9993, correspondingly. Moreover, with respect to prec_*n*_, the HBODTL-DC methodology has accessibly improved prec_*n*_ of 0.9991, whereas the DBHL, DHL-2, DHL-1, ResNet-2, TL-ResNet-2, ResNet-1, TL-RENet-1, and QSGOA-DL methodologies have reached minimal prec_*n*_ values of 0.9800, 0.9700, 0.9800, 0.9700, 0.9800, 0.9700, 0.9900, and 0.9986, correspondingly.

Figure 11 reports a accu_*y*_ comparative analysis of the HBODTL-DC algorithm with recent techniques on CXR images. The outcomes exposed that the HBODTL-DC model has gained maximal performance over other techniques. With respect to accu_*y*_, the HBODTL-DC technique has presented superior accu_*y*_ of 0.9992, whereas the DBHL, DHL-2, DHL-1, ResNet-2, TL-ResNet-2, ResNet-1, TL-RENet-1, and QSGOA-DL algorithms have reached decreased accu_*y*_ values of 0.9853, 0.9829, 0.9814, 0.9721, 0.9814, 0.9721, 0.9806, and 0.9979, correspondingly.

These results and discussion reported that the HBODTL-DC model has showcased enhanced COVID-19 classification performance over other methods.

## 5. Conclusion

In this study, a new HBODTL-DC model has been developed for the identification of COVID-19 on CXR images. The offered HBODTL-DC model includes GF preprocessing, NASNetLarge feature extraction, HBO based hyperparameter optimization, and ENN-related classification. The structure of the HBO algorithm supports ineffectual choice of hyperparameters related to the NASNetLarge model, which in turn considerably improves the classifier results. At the final stage, the ENN model receives the feature vectors as input and categorizes the CXR images into distinct classes. The experimental validation of the HBODTL-DC model takes place on the benchmark CXR image dataset, and the outcomes are reviewed under various dimensions. The experimental outcomes stated the supremacy of the HBODTL-DC model over recent approaches. Therefore, the presented HBODTL-DC model can be utilized for effectual COVID-19 classification. In the future, a multimodal DL-based fusion model can be designed to enhance the classifier results of the HBODTL-DC model [1].

## Figures and Tables

**Figure 1:** Block diagram of the HBODTL-DC technique.

**Figure 2:** Structure of the ENN.

**Figure 3:** Sample images.

**Figure 4:** Confusion matrices of HBODTL-DC technique: (a) run-1, (b) run-2, (c) run-3, (d) run-4, and (e) run-5.

**Figure 5:** Average analysis of HBODTL-DC technique: (a) run-1, (b) run-2, (c) run-3, (d) run-4, and (e) run-5.

**Figure 6:** Precision-recall curve analysis of HBODTL-DC technique.

**Figure 7:** ROC curve analysis of HBODTL-DC technique.

**Figure 8:** TA and VA analysis of the HBODTL-DC technique.

**Figure 9:** TL and VL analysis of the HBODTL-DC technique.

**Figure 10:** Comparative analysis of the HBODTL-DC technique: (a) Sens_*y*_, (b) Spec_*y*_, (c) Prec_*n*_, and (d) *F*_score_.

**Figure 11:** Accu_*y*_ analysis of the HBODTL-DC technique with existing approaches.

**Table 1:** Result analysis of the HBODTL-DC technique with various measures and runs.

Class labels	Accuracy	Precision	Sensitivity	Specificity	*F*-score
Run-1					
COVID-19	99.41	99.20	99.38	99.43	99.29
Healthy	99.24	99.53	98.64	99.67	99.08
Viral pneumonia	99.47	97.66	99.33	99.50	98.49
Average	99.38	98.80	99.12	99.54	98.95

Run-2					
COVID-19	99.51	99.32	99.50	99.52	99.41
Healthy	99.45	99.66	99.01	99.76	99.33
Viral pneumonia	99.58	98.24	99.33	99.63	98.78
Average	99.51	99.07	99.28	99.64	99.17

Run-3					
COVID-19	99.72	99.69	99.63	99.78	99.66
Healthy	99.73	100.00	99.35	100.00	99.67
Viral pneumonia	99.70	98.32	100.00	99.64	99.15
Average	99.72	99.34	99.66	99.81	99.49

Run-4					
COVID-19	99.88	99.75	99.97	99.82	99.86
Healthy	99.95	99.97	99.91	99.98	99.94
Viral pneumonia	99.94	100.00	99.63	100.00	99.81
Average	99.92	99.91	99.83	99.93	99.87

Run-5					
COVID-19	99.81	99.66	99.88	99.76	99.77
Healthy	99.87	99.88	99.81	99.91	99.84
Viral pneumonia	99.88	99.85	99.48	99.97	99.66
Average	99.85	99.80	99.72	99.88	99.76

**Table 2:** Comparative analysis of the HBODTL-DC technique with existing approaches.

Methods	Sensitivity	Specificity	Accuracy	Precision	*F*-score
DBHL	0.9900	0.9800	0.9853	0.9800	0.9800
DHL-2	0.9900	0.9700	0.9829	0.9700	0.9800
DHL-1	0.9800	0.9800	0.9814	0.9800	0.9800
ResNet-2	0.9700	0.9700	0.9721	0.9700	0.9700
TL-ResNet-2	0.9800	0.9800	0.9814	0.9800	0.9800
ResNet-1	0.9700	0.9700	0.9721	0.9700	0.9700
TL-RENet-1	0.9700	0.9900	0.9806	0.9900	0.9800
QSGOA-DL	0.9972	0.9986	0.9979	0.9986	0.9979
HBODTL-DC	0.9983	0.9993	0.9992	0.9991	0.9987

## Data Availability

No datasets were generated during the current study.
